# To Study the Effect of Individualized Nursing Model Based on MDT Concept on Limb Function Recovery and Quality of Life in Patients with Breast Cancer

This article has been retracted.

**DOI:** 10.1155/2022/1032503

**Published:** 2022-09-09

**Authors:** Yue Chen, Feng Luo, Guo Shi

**Affiliations:** Department of Breast and Thyroid Surgery, First Affiliated Hospital, Chongqing Medical University, Chongqing, China 400016

## Abstract

**Objective:**

To study the value of the individualized nursing model based on the concept of multidisciplinary team (MDT) on recovery of limb function and quality of life in patients with breast cancer.

**Methods:**

A total of 110 breast cancer patients admitted to our hospital from January 2021 to December 2021 were selected as the research objects. The 110 breast cancer patients were divided into the research group (*n* = 55) and the control group (*n* = 55) according to the random number table method. The control group received routine care. The research group implemented individualized nursing based on the MDT concept on the basis of routine nursing. The disabilities of the arm, shoulder, and hand (DASH) scores before nursing and 1 month after nursing were studied in the two groups, Hamilton anxiety scale (HAMA) score, Hamilton depression scale (HAMD) score, and Functional Assessment of Cancer Therapy-B (FACT-B) score.

**Results:**

After 1 month of nursing, the DASH score of the research group was lower than that of the control group, and the difference was statistically significant (*P* < 0.05), and after 1 month of nursing, the HAMA score of the research group was lower than that of the control group (*P* < 0.05). After 1 month of nursing, the HAMD scale score of the research group was lower than that of the control group, and the difference was statistically significant (*P* < 0.05). After 1 month of nursing, the FACT-B score of the research group was higher than that of the control group, and the difference was statistically significant (*P* < 0.05).

**Conclusion:**

The individualized nursing model based on the MDT concept has high application value for breast cancer patients. This nursing model can improve the function of limb movement, relieve the patient's anxiety and depression, and improve the patient's quality of life. This nursing model is worthy of clinical promotion.

## 1. Introduction

There are 5.7 million female breast cancer patients in the world by 2018. In China, breast cancer with 573000 confirmed number has become the most popular among women in 2018 [1]. In recent years, more and more breast cancer patients have been discovered and treated in a timelier manner because of the continuous improvement of diagnosis and treatment technology and people's health awareness with surgery as the center. The lack of breasts after surgery and various side effects of chemotherapy not only bring huge psychological pressure to patients but also seriously affect the quality of life of patients. The comprehensive treatment mode supplemented by chemotherapy, radiotherapy, and endocrine and targeted therapies has significantly improved the survival rate of breast cancer [2–5]. But shoulder joint dysfunction is still one of the most common complications of breast cancer patients [6–8].

Tumor treatment is becoming more and more complex, alone cannot meet the needs of diagnosis, treatment, and prevention of breast cancer and other tumor diseases [9–14]. The management of breast cancer patients requires the collaboration of experts in different fields. Multidisciplinary model (MDT) arises at the historic moment and gradually develops. As early as 1966, B. Fisher and E. Fisher and De Lena et al. published that breast cancer, as a systemic disease, should need comprehensive management and systemic systematic treatment in the early stage [15, 16]. MDT can establish a multidisciplinary platform for correct and rapid diagnosis of diseases, strengthening interdisciplinary communication, collecting data fully and accurately, formulating treatment plans according to evidence-based medicine. Through joint discussion, multidisciplinary experts communicate with each other timely and fully, which helps to reduce the probability of negligence in diagnosis and treatment. It is of great benefit to the improvement of the prevention, diagnosis, and treatment of breast cancer [17, 18]. Therefore, this study selected 110 breast cancer patients as the research object to detect the influence of individualized nursing model based on MDT concept on limb function recovery and quality of life of breast cancer patients.

## 2. Materials and Methods

### 2.1. General Information

A total of 110 patients with breast cancer treated from Jan. 2021 to Dec. 2021 were selected. 110 cases with breast cancer were randomly divided into the research group (*n* = 55) and the control group (*n* = 55). All patients in the research group were female, who are aged 22 to 64 years old with an average of 49.45 ± 5.16 years. Pathological classification: 30 cases of noninvasive carcinoma and 25 cases of invasive carcinoma. In the control group, all were female patients, aged 21-65 years, with an average of 49.48 ± 5.23 years. Pathological classification: 29 cases of noninvasive carcinoma and 26 cases of invasive carcinoma. There was no significant difference in general data between the two groups (*P* > 0.05).

Inclusion criteria: (1) all patients met the diagnostic criteria for breast cancer and were pathologically diagnosed as breast cancer; (2) after the researcher stated the purpose of the study, volunteer to participate in the researcher; (3) patients who would undergo axillary lymph node dissection; (4) the patients could learn to use WeChat platform for intervention feedback; and (5) clear consciousness, normal language expression, strong reading ability and unhindered communication with researchers.

Exclusion criteria: (1) mental and cognitive disorders; (2) severe heart failure, renal failure, and liver disease; (3) edema symptoms such as nephrogenic, cardiogenic, and malnutrition; and (4) bilateral breast cancer, recurrence, and other organ metastasis.

Exclusion criteria: (1) patients who did not complete all intervention and data collection and (2) the patients dropped out of the study.

### 2.2. Methods

#### 2.2.1. Technical Route

The technical route is shown in Figure 1.

#### 2.2.2. Intervention Programme

The control group received routine nursing, including admission education, preoperative preparation, diet guidance, rehabilitation exercise guidance, and discharge guidance. Patients were instructed to raise the affected limb after operation and massage the affected limb with appropriate strength. The intervention lasted for 1 month.

Research group scheme: implement individualized care based on the MDT concept on the basis of routine care. (1) Individualize nursing based on the concept of MDT. Organize a case discussion meeting once a week to communicate among team members. The nurse in charge of the bed reports the mental and physical condition of the patient, the specialist reports the operation of the patient, the rehabilitation physician, and the psychologist physicians and nutritionists are, respectively, responsible for solving the problems of patients' rehabilitation, psychology, diet, etc. (2) Establish an individualized care team based on the MDT concept. It consists of oncology specialists, tube nurses, specialist nurses, rehabilitation specialists, psychologists, nutritionists, imaging specialists, plastic surgeons, etc. The radiologists are responsible for evaluating the imaging results of patients, and specialist nurses formulate nursing plans based on the discussion content, as follows. ① Use nutritional risk screening and assessment for patients. Table (NRS-2002) is used for nutritional risk assessment. The measures for those who are sensitive to surgical fasting and fasting are that patients who are to be operated can take 1 bottle of perioperative clear drink 355 mL (surgical energy) before 12:00 after dinner before surgery. One more bottle can be taken before 6:00 in the morning for one operation. If there is no nausea and vomiting within 6 hours after the operation, a total of 1 bottle can be consumed in small amounts and multiple times. After 6 hours, normal food can be taken. ② Breast cancer patients are prone to complications such as lymphedema and skin flap necrosis after surgery. Demonstrate how to perform manual lymphatic drainage for patients and their families. The superficial lymph nodes of the back and groin should be massaged in sequence, and the scar tissue should be gently massaged along the breast surgery incision. It is advisable not to have redness after massage. After the surgical sutures were removed, the patients were required to perform manual lymphatic drainage 3 times a day, and the duration of a single session was 10 minutes. ③ Rehabilitation function training: 1-2 days after the operation, the wrist and elbow joints will be active. At the same time, the grip power ball will start to perform no more than 3 groups of 10 times a day, and the shoulder joint will be active on the third day. When the activity is above 90°, the grip strength training can be increased to 5 sets of 15-20 times per day. 7-10 days start to strengthen the shoulder joint lifting, back extension, abduction, and rotation exercises. After 14 days, you can start wall climbing exercise, ring exercise, etc. After 1 month, you can start mild resistance exercise, 2-3 times a week, with a 48-hour interval between every 2 training sessions. Under the guidance of a rehabilitation specialist, adjust the range of motion of the shoulder joint and grip strength exercises according to the patient's pain and increased drainage. Deep breathing exercises should be combined during exercise. ④After breast cancer surgery, it is easy to have low self-esteem, depression, anxiety, and other psychology disorders. Psychologists evaluate the patient's psychological state, actively talk with the patient, listen to the patient's confidence, and summarize the patient's psychological problems when listening to confidence. The causes are analyzed in depth, and then, patients are given comfort and enlightenment according to the causes. Positive suggestion, biofeedback, relaxation training, and other methods are used for psychological counseling, nurses in tube bed strengthen communication with patients, and family members and spouses are encouraged to give more support to patients.

### 2.3. Observation Indicators

1. The quality of life measurement scale (Functional Assessment of Cancer Therapy-B (FACT-B)) scores of breast cancer patients before and after nursing in the two groups were studied. The FACT-B scale [19] includes a total of 36 items in 5 areas, including four areas: physiological status, social and family status, emotional status, and functional status. Entries require reverse scoring. The total score of the scale ranges from 0 to 144 points. The higher the score, the better the quality of life in the corresponding field
2. To study the scores of Hamilton anxiety scale (HAMA), the score criteria of HAMA scale were applied to assess anxiety state [20]
3. To study the scores of Hamilton depression scale (HAMD), the score standard of HAMD scale [21] <8 means the patient is normal and has no depression; the score 8~20 means the patient has the possibility of depression; the score 21~35 means the patient must have depression; the score > 35 means the patient's depression is serious
4. The upper extremity dysfunction rating scale (disabilities of the arm, shoulder, and hand (DASH)) scores before and after nursing in the two groups were studied. The DASH scale [22] has a total of 30 questions, and each question is scored from 1 to 5. The higher the score, the more serious the dysfunction. Calculate the score according to [(total score/number of answers) − 1] × 25

### 2.4. Statistical Analysis

IBM SPSS 24.0 software was applied for statistical analysis. The measurement data were expressed by mean ± standard deviation. The counting data were expressed by frequency or rate. The *t*-test was used when measurement data obey normal distribution, and rank sum test was used when it did not obey normal distribution. The *χ*^2^ test was used to compare the classified counting data. Repeated measurement data were analyzed by repeated measurement analysis of variance. Main effect test results were used when there was no interaction, and simple effect analysis was carried out when there was interaction. *P* < 0.05 indicated that the difference between groups is statistically significant.

## 3. Results

### 3.1. The Scores of DASH Scale before Nursing and 1 Month after Nursing in Two Groups

Following one-month nursing, the score of DASH scale in the study cohort was higher than that in the control cohort, and the difference was statistically significant (*P* < 0.05). This result indicated that the DASH score of the research group was better than that of the control group. All results are shown in Table 1.

### 3.2. The Scores of HAMA Scale before Nursing and 1 Month after Nursing in Two Groups

One month after nursing, the score of HAMA scale in the research group was lower than that in the control group, and the difference was statistically significant (*P* < 0.05). This result indicated that the HAMA scores of the research group were better than those of the control group. All results are shown in Table 2.

### 3.3. The Scores of HAMD Scale in Two Groups Were Studied

Following one-month nursing, the score of HAMD scale in the research group was lower than that in the control group, and the difference was statistically significant (*P* < 0.05). This result indicated that the HAMD scale of the research group was better than that of the control group. All results are shown in Table 3.

### 3.4. The FACT-B Scores of the Two Groups Were Observed

Following one-month nursing, the FACT-B score of the research group was higher than that of the control group, and the difference was statistically significant (*P* < 0.05). This result indicated that the FACT-B scores of the research group were better than those of the control group. All results are shown in Table 4.

## 4. Discussion

The evidence has reported that for patients, MDT can effectively improve the survival rate of patients [23–31], increase patients' satisfaction [32], pay attention to patients' mental health [33], and improve the timeliness and accuracy of diagnosis [34]. For medical staff, MDT can enhance interdisciplinary communication and interaction, improve consistency in the implementation of guidelines, and provide a platform for specialist education to increase access to clinical trials. This study selected 110 breast cancer patients as the research object to detect the influence of individualized nursing model based on MDT concept on limb function recovery and quality of life of breast cancer patients.

The results of this study showed that after individualized nursing based on MDT concept, the score of DASH scale was lower than that of routine nursing, the score of HAMA and HAMD scale was lower than that of routine nursing, and the score of FACT-B was higher than that of routine nursing. It is proved that the application value of individualized nursing based on MDT concept in breast cancer patients is more significant, and it is more helpful to improve limb motor function, relieve anxiety and depression, and improve the quality of life. This is mainly because, on the one hand, breast cancer treatment will no longer belong to nurses but to the entire breast cancer treatment team.

Breast cancer MDT team experts include breast surgery, oncology, pathology, imaging (ultrasound, mammography, magnetic resonance, and nuclear medicine), radiotherapy, and breast specialist nurses. The UK Department of Health defines MDT as “experts from different medical fields discuss patients' treatment decisions together at a specific time and place (or by remote/video or teleconference) and each expert can make diagnosis and treatment decisions about patients independently.” According to the specific situation, it can include drug therapists, geneticists, physiotherapists, psychologists, plastic surgeons, dietitians, and social workers [35, 36]. This study introduces the concept of multidisciplinary teamwork, in which breast cancer specialist nurses play a leading role, and imaging technologists, oncologists, and pharmacists assume different responsibilities in the team. When specialist nurses encounter problems that cannot be dealt with alone, they contact team members for multidisciplinary consultation and discussion. Members of different disciplines perform their own functions, complement each other, and formulate standardized and targeted diagnosis and treatment plans so that various disciplines integrate and promote each other and reach a consensus on treatment methods and ideas. It has improved the medical risk prevention ability of specialist nurses and improved the nursing quality of breast cancer patients.

Secondly, the members of the individualized nursing group based on the concept of MDT cooperate with each other and give patients professional, standardized, and systematic nursing intervention, which can improve the nursing quality and improve the prognosis of patients. Its purpose is to transform the traditional empirical therapy into modern teamwork therapy and individualized therapy [37, 38]. First of all, on the premise of accurate diagnosis, the diagnosis process of patients usually includes the first clinical consultation of patients, the improvement of imaging examination, the final pathological diagnosis of tumor puncture, and the formulation of individual treatment plan according to the specific condition of the patient. Specifically, breast cancer patients after routine examination, by imaging doctors, to judge the specific condition of upper limb dysfunction, upper limb edema and other symptoms, by the MDT team to formulate a nursing plan, under the guidance of the MDT team for treatment and nursing, until the upper limb edema symptoms are eliminated, so as to correct the condition of upper limb dysfunction and improve the quality of life [39, 40].

Third, MDT explores disease treatment strategies by establishing a multidisciplinary platform, taking people as the fundamental principle, and relying on team members of various disciplines, rather than the traditional form of “disease-centered.” Specifically, in the intervention, rehabilitation physicians instruct patients to exercise upper limb function, which can effectively improve limb function. Psychologists evaluate the psychological state of patients in time, devote themselves to solving the actual psychological problems of patients, use positive suggestion, biofeedback, relaxation training, and other methods for psychological counseling, and strengthen communication between nurses and patients. Encouraging family members and spouses to give more support to patients can effectively alleviate patients' anxiety and depression, make patients have more confidence in treatment, and improve patients' compliance. This study still has some shortcomings. Firstly, the quality of this study is limited due to the small sample size we included in the study. Secondly, this research is a single-center study and our findings are subject to some degree of bias. Therefore, our results may differ from those of large-scale multicenter studies from other academic institutes. This research is still clinically significant and further in-depth investigations will be carried out in the future.

To sum up, the individualized nursing model based on the MDT concept has high application value for breast cancer patients. This nursing model can improve the function of limb movement, relieve the patient's anxiety and depression, and improve the patient's quality of life. This nursing model is worthy of clinical promotion.

## Figures and Tables

**Figure 1:** Technical route.

**Table 1:** The DASH score of two groups before nursing and 1 month after nursing.

Grouping	Before nursing	After one month of nursing
Control group	75.54 ± 2.19	41.82 ± 1.11^∗^
Research group	75.55 ± 2.12	25.69 ± 1.03^∗^
*tvalue*	0.024	78.998
*Pvalue*	0.981	0.000

Note: ∗ represents that after one month of nursing in this group, compared with that before nursing, *P* < 0.05.

**Table 2:** The HAMA scores of the two groups before nursing and 1 month after nursing.

Grouping	Before nursing	After one month of nursing
Control group	8.45 ± 1.33	6.59 ± 1.17^∗^
Research group	8.51 ± 1.29	4.08 ± 0.15^∗^
*tvalue*	0.240	15.781
*Pvalue*	0.811	0.000

Note: ∗ represents that after one month of nursing in this group, compared with that before nursing, *P* < 0.05.

**Table 3:** The score of HAMD scale before nursing and 1 month after nursing in two groups.

Grouping	Before nursing	After one month of nursing
Control group	10.89 ± 2.12	7.32 ± 1.22^∗^
Research group	10.92 ± 2.09	6.11 ± 0.13^∗^
*tvalue*	0.075	7.314
*Pvalue*	0.941	0.000

Note: ∗ represents that after one month of nursing in this group, compared with that before nursing, *P* < 0.05.

**Table 4:** The FACT-B scores of the two groups prenursing and after 1-month nursing.

Grouping	Before nursing	After one month of nursing
Control group	60.39 ± 2.84	77.09 ± 4.33^∗^
Research group	60.44 ± 2.77	85.17 ± 3.04^∗^
*tvalue*	0.093	11.326
*Pvalue*	0.926	0.000

Note: ∗ represents that after one month of nursing in this group, compared with that before nursing, *P* < 0.05.

## Data Availability

The datasets used and analyzed during the current study are available from the corresponding author upon reasonable request.
